The article "Risk Factors of Cerebral Infarction and Myocardial Infarction after Carotid Endarterectomy Analyzed by Machine Learning" was published in 2020. Journal: Comput Math Methods Med.

# Risk Factors of Cerebral Infarction and Myocardial Infarction after Carotid Endarterectomy Analyzed by Machine Learning

**DOI:** 10.1155/2020/6217392

**Published:** 2020-11-12

**Authors:** Peng Bai, Yang Zhou, Yuan Liu, Gang Li, Zhengqian Li, Tao Wang, Xiangyang Guo

**Affiliations:** ^1^Department of Anesthesiology, Peking University Third Hospital, Peking University Health Science Center, Beijing, China; ^2^College of Chemistry and Molecular Engineering, Peking University, Beijing, China; ^3^Department of Neurosurgery, Peking University Third Hospital, Peking University Health Science Center, Beijing, China

## Abstract

**Objective:**

The incidence of cerebral infarction and myocardial infarction is higher in patients with carotid endarterectomy (CEA). Based on the concept of coprotection of heart and brain, this study attempts to screen the related factors of early cerebral infarction and myocardial infarction after CEA with the method of machine learning to provide clinical data for the prevention of postoperative cerebral infarction and myocardial infarction.

**Methods:**

443 patients who received CEA operation under general anesthesia within 2 years were collected as the research objects. The demographic data, previous medical history, degree of neck vascular stenosis, blood pressure at all time points during the perioperative period, the time of occlusion, whether to place the shunt, and the time of hospital stay, whether to have cerebral infarction and myocardial infarction were collected. The machine learning model was established, and stable variables were selected based on single-factor analysis.

**Results:**

The incidence of cerebral infarction was 1.4% (6/443) and that of myocardial infarction was 2.3% (10/443). The hospitalization time of patients with cerebral infarction and myocardial infarction was longer than that of the control group (8 (7, 15) days vs. 7 (5, 8) days, *P* = 0.002). The stable related factors were screened out by the xgboost model. The importance score (*F* score) was as follows: average arterial pressure during occlusion was 222 points, body mass index was 159 points, average arterial pressure postoperation was 156 points, the standard deviation of systolic pressure during occlusion was 153 points, diastolic pressure during occlusion was 146 points, mean arterial pressure after entry was 143 points, systolic pressure during occlusion was 121 points, and age was 117 points.

**Conclusion:**

Eight factors, such as blood pressure, body mass index, and age, may be related to the postoperative cerebral infarction and myocardial infarction in patients with CEA. The machine learning method deserves further study.

The article "Risk Factors of Cerebral Infarction and Myocardial Infarction after Carotid Endarterectomy Analyzed by Machine Learning" was published in 2020. Journal: Comput Math Methods Med.

## 1. Introduction

Carotid endarterectomy (CEA) can correct the stenosis of the common carotid artery or internal carotid artery and prevent stroke by removing the atherosclerotic plaque. The major complications after CEA include cerebral infarction and myocardial infarction; the incidence rate of cerebral infarction is reported as 3% to 4% [1, 2], and the incidence of myocardial infarction is 0.5%-1% [3]. Because of the particularity of the operation site and perioperative management of CEA, which is based on the concept of cardio cerebral coprotection in the world, the risk factors of cerebral infarction, myocardial infarction, and other events are analyzed in a unified way after they are combined, trying to find a perioperative management strategy that takes into account the cerebral and cardiac blood flow perfusion [4–6].

For the events with low incidence, the traditional statistical methods have some limitations. Machine learning is a new tool to explore and analyze big data in the field of artificial intelligence (AI), which enables computers to learn automatically and make adjustments according to the situation without human intervention or assistance. At present, the application of machine learning in clinical medicine has been preliminarily discussed [7].

In this retrospective study, the patients who underwent elective carotid endarterectomy were selected, and cerebral infarction and myocardial infarction were taken as the endpoint observation indicators. Based on the single-factor analysis, a machine learning model was established, and the relevant indicators of cerebral infarction and myocardial infarction were discussed.

## 2. Materials and Methods

### 2.1. Materials

All patients who received standard carotid endarterectomy under general anesthesia in two years were retrospectively collected as two different surgical units of the Peking University Third Hospital. Patients with CEA+CABG at the same time were excluded, and the preoperative demographic data and past medical history of the patients were collected. Because the CEA operation in our hospital is selective, all patients met the inclusion criteria for elective surgery. Patients with hypertension were regularly taking diuretics, calcium antagonists, ACEI, or ARB drugs to control blood pressure before the operation, and the patients with diabetes mellitus were satisfied with preoperative blood glucose control. Patients with poor blood pressure or blood glucose control would first receive specialist medical treatment before meeting the criteria for elective surgery. All patients received the cervical vascular ultrasound and/or CTA before the operation. According to NASCET criteria, the degree of cervical vascular stenosis was divided into mild (0%-49%), moderate (50%-69%), and severe stenosis and occlusion (70% and above). The systolic, diastolic, and mean arterial pressures of one day before operation (T1), entering the operating room (T2), the 10 minutes before carotid occlusion (T3), the period during occlusion (T4), the 10 minutes after blood flow recovery (T5), and one day after the operation (T6) were recorded. The blood pressure during the occlusion (T4) was recorded once every 5 minutes and with the average value of blood pressure during each patient's occlusion as the blood pressure during the period of occlusion (T4). And record the blood pressure standard deviation during the occlusion. Record the time of carotid artery occlusion, whether to use the shunt, and hospitalization after the operation, whether cerebral infarction (definite neurological symptoms, imaging examination confirmed that there were new infarcts or the area of original infarcts increased) or myocardial infarction (myocardial ischemia symptoms and laboratory examination indicated that myocardial injury markers were increased and confirmed by consultation of cardiology department) occurred during hospitalization.

The article "Risk Factors of Cerebral Infarction and Myocardial Infarction after Carotid Endarterectomy Analyzed by Machine Learning" was published in 2020. Journal: Comput Math Methods Med.

Standard carotid endarterectomy was performed by surgeons in both surgical units. However, there were different strategies for the selection of shunt. In one surgical unit, the surgeon decided whether to place the carotid shunt according to the results of preoperative angiography or CTA: if the imaging results showed that the contralateral carotid artery was severely stenosis or occlusion and the Willis ring was incomplete (the definition of Willis ring incomplete is that CTA shows any part of the ring, which is composed of a bilateral anterior cerebral artery, the initial segment of a bilateral posterior cerebral artery, end of the bilateral internal carotid artery, and anterior and posterior communicating arteries that cannot be developed) and the anterior or posterior communicating arteries were not opened satisfactorily, the shunt was placed during the operation, which was called the imaging group. In the other surgical unit, the surgeon did not require angiography or CTA preoperation. The surgeon measured stump pressure when the carotid artery was occluded. If the stump pressure was less than 40, a shunt would be performed, while the blood pressure is raised to meet the needs of cerebral perfusion when the stump pressure is greater than or equal to 40 mmHg. These patients were called the stump pressure group.

The results of our previous studies suggest that different bypass strategies are not risk factors for postoperative severe adverse events. Therefore, different bypass strategies are included in the machine learning model as a related factor. Cerebral infarction and myocardial infarction during hospitalization were taken as observation indexes. Patients with cerebral infarction and/or myocardial infarction were defined as the event group in this study, and those who did not occur were defined as the control group.

The article "Risk Factors of Cerebral Infarction and Myocardial Infarction after Carotid Endarterectomy Analyzed by Machine Learning" was published in 2020. Journal: Comput Math Methods Med.

### 2.2. Statistical Methods

SPSS 23.0 was used for the analysis of the data. The measurement data conforming to the normal distribution were expressed by mean ± standarddeviation ($\bar{x}\pm \text{SD}$). Independent sample *t*-test is used for analysis. Data that do not conform to normal distribution are represented by median and quartile, and the Wilcoxon rank-sum test is used for analysis. Counting data are tested by the chi-square test or Fisher exact probability method. *P* < 0.05 was statistically significant.

### 2.3. Machine Learning

*Model building*: the widely used tool kit scikit-learn 0.21 (https://scikit-learn.org/stable/) [8] was used to conduct algorithm screening for the two classification problems represented in this study. The algorithms included in scikit-learn include linear support vector machine, decision tree, random forest, artificial neural network, quadratic discriminant analysis, and xgboost. The goal outcome was whether there was cerebral infarction and myocardial infarction during postoperative hospitalization. All characteristic parameters of all patients were included in the model, and the accuracy of the positive results screened by different algorithms was taken as the evaluation standard, and the model with the highest accuracy was selected.

*Cross-validation optimization prediction model*: used as the selected model. Each time, 3/4 of the data were randomly extracted from the positive samples (event group) and the negative samples (control group) to build a training set, and the remaining 1/4 of the positive and negative samples were used as the verification set to test the model. Repeat the above steps 1000 times, and finally average the test results to balance the random error in the process of sample extraction.

*Screening stable variables*: if the AUC of the model was low or unstable after cross-validation, screen the stability of variables. Try to delete the variables with low importance score and bring the remaining variables into the model for training again. If the type and ranking order of the variable in the result did not change much when the variable was deleted, the variable was considered to have less impact on the outcome. And it was going to be deleted. If the type and ranking of the variable in the result changed a lot, the variable was considered to have a greater impact on the outcome. It was going to be retained. This was repeated until the variable can no longer be deleted. At this time, the remaining variables were the key variables that have a stable impact on the outcome.

The article "Risk Factors of Cerebral Infarction and Myocardial Infarction after Carotid Endarterectomy Analyzed by Machine Learning" was published in 2020. Journal: Comput Math Methods Med.

*The solution to the problem of unbalanced data*: when the number of cases of different types of training set data varies greatly, it is called unbalanced data. The problem was solved by adjusting the scale_pos_weight and increasing the learning rate of a small number of samples.

*Predictive variable importance score* (*Fscore*): in the process of training, variable importance score was the score of each feature given according to the number of times the variable was used as the partition variable, indicating the importance of each feature to the model. The higher score of the variable, the greater the influence of the variable on the outcome.

## 3. Results

A total of 443 cases of CEA operations under general anesthesia were included. There were 6 cases of cerebral infarction (1.4%), 10 cases of myocardial infarction (2.3%), and 16 cases of patients in the event group. There were 427 patients in the control group, of which 5 patients had carotid artery stenosis less than 50%, which did not reach the recognized surgical indications. These five patients were all severe stenosis of the contralateral carotid artery. After surgery, the patients insisted on dealing with the potential risks, so they still underwent surgical treatment. There was no significant difference in baseline data such as patients' condition, gender, age, body mass index, the incidence of previous comorbidities, and the grade of vascular stenosis (Table 1).

The single-factor analysis of blood pressure at each time point of the patients, occlusion time, bypass time during the operation, and the hospitalized time postoperation was shown in Table 2. There was no significant difference in systolic pressure (SBP), diastolic pressure (DBP), and mean arterial pressure (MBP) between the event group and the control group (*P* > 0.05). The postoperative hospital stay was 8 (7, 15) days in the event group and 7 (5, 8) days in the control group. There was a significant difference between the two groups (*P* = 0.002).

Inputted the data into machine learning, xgboost had the highest accuracy of positive events screened out by different algorithms. So xgboost was selected as the machine learning algorithm of this study (Figure 1).

In cross-validation, the AUC fluctuated between 0.2-0.9 with different random sampling. It suggested that the prediction of the model was not stable. So further evaluation of the stability of different variables on the outcome was performed to get key variables. In the beginning, all the 37 variables were put into machine learning, and the influence of variables on the outcome was evaluated according to the importance score in Table 3.

The article "Risk Factors of Cerebral Infarction and Myocardial Infarction after Carotid Endarterectomy Analyzed by Machine Learning" was published in 2020. Journal: Comput Math Methods Med.

After the selection of variables' stability, eight stable key variables were obtained: mean arterial pressure during occlusion (T4 MBP), body mass index (BMI), mean arterial pressure after the operation (T6 MBP), the standard deviation of systolic pressure during occlusion (T4 SBP standard deviation), diastolic pressure during occlusion (T4 DBP), mean arterial pressure in the operating room (T2 MBP), systolic pressure during occlusion (T4 SBP), and age. And their *F* scores were shown in Figure 2.

## 4. Discussion

Among 443 patients with CEA, 6 cases (1.4%) had cerebral infarction, which was lower than the incidence of 3%~4% reported. It might be related to the shorter observation time (hospitalization vs. 30 days postoperation). 10 cases (2.3%) of myocardial infarction were similar to the results of the Crest and Sapphire Trial (2.3%-5.9%) [9, 10]. Because of the pathophysiological changes of cardiovascular and cerebrovascular diseases, the coprotection of the heart and brain during the perioperative period of CEA had always been the focus of attention. As we all know, vascular factors such as atherosclerosis were systemic diseases, which often involved multiple organs in the whole body. It showed that patients were often accompanied by lesions in multiple parts such as the coronary artery and lower extremity artery when the carotid artery was involved. The results of Steinvil et al. [5] and Hallerstam et al. [6] indicated that the severity of carotid artery stenosis had a clear correlation with the degree of coronary artery stenosis and myocardial hypoperfusion. And previous studies had shown that cerebral infarction and myocardial infarction after CEA had many same risk factors, including age, diabetes, cardiac insufficiency, renal insufficiency, and hypotension [4, 11–15]. It was suggested that there might be a common pathophysiological basis and mechanism for the occurrence of cerebral infarction and myocardial infarction in patients undergoing CEA. Therefore, referring to the research of Gates et al. [4], this study took cerebral infarction and myocardial infarction as the research endpoint, which is based on the mechanism of cardiovascular and cerebrovascular comorbidity and the perspective of the overall prognosis of patients. It was going to explore the strategy of perioperative coprotection of heart and brain, which may provide a comprehensive and balanced optimization scheme for the perioperative management of CEA, and avoid the injury to one organ due to protecting another.

The article "Risk Factors of Cerebral Infarction and Myocardial Infarction after Carotid Endarterectomy Analyzed by Machine Learning" was published in 2020. Journal: Comput Math Methods Med.

For the events with a small sample size and low incidence, traditional statistical methods have some limitations. Compared with the traditional regression analysis, the machine learning algorithm has the advantages of loose data distribution requirements, a variety of algorithms that can be selected according to the characteristics of data, multiple random selections of samples for training, and sample error that can be balanced. The use of machine learning in the field of clinical medicine has begun [16]. Xgboost is a kind of gradient lifting algorithm in machine learning. It allocates the weight of data points with low accuracy in each round of training and finally highlights the weight of the decision tree with high classification quality to improve the accuracy and generalization ability of the algorithm [17–19]. In some research, xgboost was superior to traditional logistic regression. In this study, xgboost got the highest accuracy in the process of algorithm selection, so the subsequent data calculation was carried out by this algorithm. However, in the course of optimizing the prediction model, it was found that the efficiency of the model fluctuates greatly, which might be due to the small number of positive samples, resulting in the poor prediction efficiency of the model. Therefore, variables that have a stable impact on the predicted outcome were explored. In the process of increasing and decreasing the variables with low importance score, the 8 variables always ranked in the top 8 and could not be excluded, including mean arterial pressure during occlusion, body mass index, mean arterial pressure after the operation, the standard deviation of systolic pressure during occlusion, diastolic pressure during occlusion, mean arterial pressure entering the room, systolic pressure during occlusion, and age. And the order of these 8 variables only changes within one or two. It was suggested that no matter how large the error caused by random sampling was, these 8 factors always had a stable effect on the outcome. In this study, the sample size was small and the incidence rate was low. The limited number of factors that can be incorporated into traditional logistic regression leads to limited analysis. It provided a new way to explore the related factors of cardiac and cerebral complications after CEA by using machine learning.

Among the eight key variables obtained by machine learning, six were related to blood pressure, including systolic pressure, diastolic pressure, and mean arterial pressure. For cerebral infarction, many previous studies had reported the relationship between systolic blood pressure and cerebral infarction, and it was considered that systolic blood pressure was a risk factor with predictive value for cerebral infarction [20–22]. In recent years, some studies had reported the predictive value of diastolic blood pressure in perioperative cerebral infarction. The results of de Waard et al. [23] showed that high diastolic pressure (>90 mmHg) was an independent risk factor for perioperative cerebral infarction and death (or = 2.06, 95% CI 1.04-4.06, and *P* = 0.04). The mean arterial pressure, as a factor affecting cerebral perfusion directly, was also of great significance. In terms of time, it included the distribution of three-time points: preoperation, intraoperative, and postoperation. ICSS Research (International Cardioid Stenting Study) pointed out that preoperative blood pressure was an independent risk factor for myocardial infarction and death after operation [24]. In terms of intraoperative management, intraoperative blood pressure management has always been the core of anesthesia management in CEA. The results of this study suggested that the mean arterial pressure, the standard deviation of systolic blood pressure, diastolic blood pressure, and systolic blood pressure during occlusion were all of high importance in classification decision-making, with important weight. So we should focus on the influence of blood pressure (including mean arterial pressure, systolic blood pressure, and diastolic blood pressure) on early postoperative cerebral infarction.

The article "Risk Factors of Cerebral Infarction and Myocardial Infarction after Carotid Endarterectomy Analyzed by Machine Learning" was published in 2020. Journal: Comput Math Methods Med.

But at the same time, we also noticed that the machine learning method in this study did not get a stable prediction model, but a stable influencing factor was obtained in the stability screening of related factors, suggesting that although blood pressure has an important impact on the outcome, it is not an independent determinant. There may be other factors not included in this study, which may also play an important role, such as the use of antiplatelet drugs before the operation and embolic shedding caused by embolism. It has been reported that microemboli detachment is one of the most important factors of stroke during the perioperative period of CEA [25]. And the use of antiplatelet drugs will reduce the incidence of stroke in patients after CEA [26]. In this study, due to the limitations of retrospective study data, microemboli, preoperative antiplatelet drug use, and other factors were not included. Whether the addition of other factors will change the results of machine learning remains to be further verified by future research.

Previous studies had shown that there was a correlation between hypotension and myocardial infarction, but there was no clear consensus on the definition of the degree and duration of hypotension in different studies [15, 27]. In this study, the importance score of systolic blood pressure standard deviation in the period of occlusion was in the fourth place, indicating that besides the high and low levels of blood pressure, the fluctuation degree of systolic blood pressure was also of great significance. The results of Mutch et al. showed that patients with high blood pressure fluctuation during the operation were more likely to suffer from myocardial ischemia [28]. It was suggested that the mechanism of postoperative myocardial infarction was complex, and the level of blood pressure might not be an independent predictor. Many other factors that affect the myocardial oxygen balance should be considered comprehensively, including the degree of blood pressure fluctuation, heart rate, and systolic force.

The article "Risk Factors of Cerebral Infarction and Myocardial Infarction after Carotid Endarterectomy Analyzed by Machine Learning" was published in 2020. Journal: Comput Math Methods Med.

BMI was in the second place of importance score and age was in the eighth. The effect of body weight index remained controversial. The previous view showed that overweight or obesity was the main related factor of vascular diseases and might shorten the median survival time by 2-4 years [29]. However, some studies showed that patients with BMI of 30-35 kg·m^−2^ had higher survival rates [30] and lower stroke rates [31] for CEA. The effect of BMI on CEA may come from the deeper mechanism which needs further study. Previous studies reported that age was a common risk factor for cerebral infarction and myocardial infarction after CEA [4, 12],

In this study, the data with small sample size and low incidence rate was analyzed by the machine learning method, which was limited by traditional logistic regression analysis. In the case of the poor stability of the model, the stability of the relevant factors was explored to screen the relevant factors as a new attempt. The application of these methods needs more study in the future. And this method can not give the direct impact of specific factors on the outcome, although the selected risk factors are consistent with the previous reports. The optimal perioperative management of CEA needs more study.

## 5. Conclusion

Eight factors were screened out by machine learning method, which may be related to early cerebral infarction and myocardial infarction after CEA, including mean arterial pressure during occlusion, body mass index, mean arterial pressure postoperation, the standard deviation of systolic pressure during occlusion, diastolic pressure during occlusion, mean arterial pressure entering the room, systolic pressure during occlusion, and age. The application of the machine learning method in clinical research deserves further study in the future.

The article "Risk Factors of Cerebral Infarction and Myocardial Infarction after Carotid Endarterectomy Analyzed by Machine Learning" was published in 2020. Journal: Comput Math Methods Med.

## Figures and Tables

**Figure 1:** Accuracy of machine learning algorithms.

**Figure 2:** Variables and importance (the higher the *F* score, the greater impact on the outcome). T1: preoperative; T2: entering operating room; T3: 10 minutes before carotid occlusion; T4: during occlusion; T5: 10 minutes after blood flow recovery; T6: one day after operation.

**Table 1:** Baseline characteristics of the patients.

Variable	Event group (*n* = 16)	Control group (*n* = 427)	*P*
Male sex-no. (%)	14 (87.5%)	337 (78.9%)	0.605
Age (yr)	66.0 (62.3, 76.5)	66.0 (61.0, 72.0)	0.301
BMI (kg∙m^−2^)	25.3 (22.3, 27.6)	24.7 (22.8, 27.2)	0.749
Hypertension-no. (%)	11 (68.8%)	315 (73.8%	0.874
Diabetes mellitus-no. (%)	6 (37.5%)	151 (35.4%)	0.861
Coronary heart disease-no. (%)	6 (37.5%)	127 (29.7%)	0.699
Preoperative neurological symptoms infarction-no. (%)	6 (37.5%)	142 (33.3%)	0.833
TIA-no. (%)	3 (18.8%)	70 (16.4%)	
No symptoms-no. (%)	7 (43.8%)	215 (50.4%)	
Carotid stenosis ipsilateral			0.365
Mild-no. (%)	0 (0.0%)	5 (1.2%)	
Moderate-no. (%)	0 (0.0%)	50 (11.7%)	
Severe-no. (%)	16 (100.0%)	372 (87.1%)	
Carotid stenosis contralateral			0.170
Mild-no. (%)	7 (43.8%)	268 (62.8%)	
Moderate-no. (%)	6 (37.5%)	80 (18.7%)	
Severe-no. (%)	3 (18.8%)	79 (18.5%)	
Vertebral stenosis ipsilateral			1.000
Mild-no. (%)	14 (87.5%)	359 (84.1%)	
Moderate-no. (%)	1 (6.3%)	23 (5.4%)	
Severe-no. (%)	1 (6.3%)	45 (10.5%)	
Vertebral stenosis contralateral			0.655
Mild-no. (%)	14 (87.5%)	358 (83.8%)	
Moderate-no. (%)	0 (0.0%)	30 (7.0%)	
Severe-no. (%)	2 (12.5%)	39 (9.1%)	
Unit			0.084
Imaging group-no. (%)	13 (81.3%)	255 (59.7%)	
Stump pressure group-no. (%)	3 (18.7%)	172 (40.3%)	

BMI: body mass index.

**Table 2:** Blood pressure during operation and postoperation of the patients.

Variable	Event group (*n* = 16)	Control group (*n* = 427)	*P*
T1 SBP (mmHg)	130 (130, 136)	130 (130, 140)	0.741
T1 DBP (mmHg)	73 (70, 78)	75 (70, 80)	0.381
T1 MBP (mmHg)	93 (90, 97)	93 (90, 98)	0.500
T2 SBP (mmHg)	163 (146, 178)	156 (145, 167)	0.246
T2 DBP (mmHg)	85 (71, 90)	80 (70, 85)	0.263
T2 MBP (mmHg)	111 (98, 118)	105 (97, 112)	0.151
T3 SBP (mmHg)	130 (120, 150)	135 (123, 147)	0.387
T3 DBP (mmHg)	62 (57, 74)	65 (60, 70)	0.479
T3 MBP (mmHg)	87 (74, 97)	90 (83, 97)	0.446
T4 SBP (mmHg)	159 ± 12	157 ± 16	0.629
T4 SBP standard deviation (mmHg)	6 (3, 9)	5 (3, 7)	0.422
T4 DBP (mmHg)	71 (66, 83)	71 (64, 78)	0.666
T4 DBP standard deviation (mmHg)	3 (2, 5)	3 (2, 4)	0.384
T4 MBP (mmHg)	101 ± 11	100 ± 10	0.634
T5 SBP (mmHg)	135 (130, 141)	130 (121, 140)	0.272
T5 DBP (mmHg)	60 (58, 73)	62 (56, 70)	0.977
T5 MBP (mmHg)	87 (79, 93)	85 (80, 92)	0.642
T6 SBP (mmHg)	140 (131, 150)	135 (130, 140)	0.160
T6 DBP (mmHg)	80 (70, 80)	75 (70, 80)	0.489
T6 MBP (mmHg)	98 (90, 103)	95 (90, 100)	0.220
Occlusion time (min)	25.0 (25.0, 30.0)	26.0 (25.0, 35.0)	0.406
Shunt-no. (%)	1 (6.3%)	45 (10.5%)	0.715
Postoperative hospital stay (day)	8 (7, 15)	7 (5, 8)	0.002^∗^

T1: preoperative; T2: entering operating room; T3: 10 minutes before carotid occlusion; T4: during occlusion; T5: 10 minutes after blood flow recovery; T6: one day after operation.

The article "Risk Factors of Cerebral Infarction and Myocardial Infarction after Carotid Endarterectomy Analyzed by Machine Learning" was published in 2020. Journal: Comput Math Methods Med.

**Table 3:** Importance weight of variables predicted by xgboost.

Number	Variable	Importance	Number	Variable	Importance
1	T4 MBP	0.239	14	Occlusion time	0.108
2	T4 SBP	0.223	15	Weight	0.095
3	T6 MBP	0.183	16	Carotid stenosis ipsilateral	0.086
4	T2 MBP	0.169	17	Carotid stenosis contralateral	0.063
5	Age	0.165	18	Vertebral stenosis contralateral	0.056
6	T3 MBP	0.160	19	Vertebral stenosis ipsilateral	0.052
7	T4 DBP	0.158	20	Diabetes mellitus	0.034
8	Height	0.142	21	Preoperative neurological symptoms	0.023
9	T4 DBP standard deviation	0.131	22	Occlusion time	0.018
10	T1 MBP	0.126	23	Coronary heart disease	0.009
11	BMI	0.120	24	Hypertension	0.009
12	T4 SBP standard deviation	0.115	25	Gender	0.005
13	T5 MBP	0.108	26	Shunt	0.002

T1: preoperative; T2: entering operating room; T3: 10 minutes before carotid occlusion; T4: during occlusion; T5: 10 minutes after blood flow recovery; T6: one day after operation.

## Data Availability

The data used to support the findings of this study are available from the corresponding author upon request.
